# Enhancing Text Generation via Parse Tree Embedding

**DOI:** 10.1155/2022/4096383

**Published:** 2022-06-10

**Authors:** Dagao Duan, Qiuli Zhang, Zhongming Han, Haitao Xiong

**Affiliations:** ^1^School of International Economics and Management, Beijing Technology and Business University, Beijing 100048, China; ^2^School of Computer Science and Engineering, Beijing Technology and Business University, Beijing 100048, China

## Abstract

Natural language generation (NLG) is a core component of machine translation, dialogue systems, speech recognition, summarization, and so forth. The existing text generation methods tend to be based on recurrent neural language models (NLMs), which generate sentences from encoding vector. However, most of these models lack explicit structured representation for text generation. In this work, we introduce a new generative model for NLG, called Tree-VAE. First it samples a sentence from the training corpus and then generates a new sentence based on the corresponding parse tree embedding vector. Tree-LSTM is used in collaboration with the Stanford Parser to retrieve sentence construction data, which is then used to train a conditional discretization autoencoder generator based on the embeddings of sentence patterns. The proposed model is extensively evaluated on three different datasets. The experimental results proved that the proposed model can generate substantially more diverse and coherent text than existing baseline methods.

## 1. Introduction

Text generation is an important foundation for many Natural Language Processing (NLP) tasks, including machine translation, summarization, and dialogue systems [1–7]. In these tasks, most of the models are based upon the sequence-to-sequence and recurrent neural network architectures, encoding the source text to a dense vector and decoding the vector to target text by maximizing the likelihood of ground-truth word given prior observed words [8, 9]. However, most of these methods lack explicit structural representation of text to generate semantically meaningful and diverse sentences [10].

Despite being widely applied, conventional text generative models tend to repeatedly generate text in the training dataset and lack the ability to create novel sentences. At the same time, naive strategies to increase diversity have been shown to compromise grammaticality [11]. The major reason is that recurrent neural language models (NLMs) lack the inductive bias to faithfully represent the full diversity of complex utterances. Indeed, it is difﬁcult for decoder to create novel and meaningful texts from scratch. The overestimation of existing texts encourages the model to copy the original sentence, which makes the generated text tend to be repeated and worthless.

To address this issue, we suggest a new text generating paradigm, called Tree-VAE. Its purpose is to convert a variable-length text into a fixed-length vector. The input sequence is mapped to a fixed-sized vector, which will then be fed to a SoftMax layer for categorization or other tasks. The proposed model consists of a pretrained parse tree encoder that is responsible for generating embedding of text structure, a text encoder that encodes the source text to a dense vector representation, and a decoder that generates realistic sentences from arbitrary latent vector and corresponding parse tree embedding. In this paper, we consider that the text parse tree embedding is a structural condition for producing diversiﬁed text by the decoder. In training learning stage, text in the corpus will be parsed into syntactic tree by the Stanford dependency parser and then encoded into parse tree embedding vector with Tree-LSTM parse encoder [10, 12]. The parse tree encoder can assign similar vectors for texts with similar structures. Then, the parse tree embedding vector is fed into the decoder, which encourages the decoder to produce coherent and structurally similar text. The advantage is that the structure features of text from the corpus provide a high-quality starting point: they are grammatical and naturally diverse. The decoder then generalizes the structure properties to novel sentences.

In parse tree encoder pretraining, given a sentence, we ﬁrst parse it to syntactic tree and remove word content, only keeping part of speech for each node in the tree, followed by encoding the structure tree to a dense vector. To generate similar structural embedding vector for most structurally similar sentences, we build a standard hierarchical LSTM responsible for reconstructing the original structure tree [13]. Attention mechanism is used for this hierarchical LSTM network. We train the parse tree encoder and LSTM network by maximizing an approximation to the reconstructed log-likelihood. We employ parse tree encoder architecture like autoencoding, extending it to encode structure features of text. A good parse tree encoder extracts the rich information from the structure tree and increases quality of outputs for decoder.

Contrary to existing works which generate from scratch, the core of our model is a parse tree encoder composed of Stanford dependency parser and Tree-LSTM layers. This choice of architecture helps to gain more text structure information, which is crucial for generating high-quality text. The analysis of the experimental results shows that our parse tree encoder can effectively encode text structure and improve the performance of the decoder.

Our contributions are listed as follows:

- We propose a new model, called Tree-VAE, which generates diversiﬁed and grammatical text conditioned on text structure features.
- We propose a novel parse tree encoder, which can extract the rich information from the structure tree and assign similar structural embedding vector for most structurally similar sentences.
- The experimental results on text generation task show that our method can generate more coherent and informative text compared to existing methods.

## 2. Related Work

Currently, there are two major streams of approaches to text generation modeling: the variational autoencoder and generative adversarial networks [14–16].

GAN has been demonstrated to be eﬀective in the computer vision domain but has not shown signiﬁcant improvement in NLP community. The reason is that, in GANs, the text sequences are evaluated as the discrete tokens whose values are nondifferentiable, which makes it difﬁcult to train. To tackle this problem, SeqGAN addressed this issue by the policy gradient inspired from the reinforcement learning [17, 18]. RankGAN learned model from the relative ranking information between the machine-written and the human-written sentences in an adversarial framework and relaxed the training of the discriminator to a learning-to-rank optimization problem [19]. Mali-GAN [20] modiﬁes the original GAN objective and proposes a set of training techniques to reduce the potential variance [12].

Another problem for the adversarial sequence generation models is that the binary feedback from the discriminator is not sufﬁciently informative. Leak-GAN allowed the discriminative network to leak its own high-level extracted features to the generative network to further help the guidance [21]. The generator incorporates such informative signals into all generation steps through an additional MANAGER module, which takes the extracted features of current generated words and outputs a latent vector to guide the WORKER module for next word generation. DP-GAN assigned low reward for repeated text and high reward for novel text, encouraging the generator to produce diverse and informative text [22].

The variational autoencoder is a generative model based on classical autoencoder [14, 23–26]. There are some research that deal with text generation problem within the VAE framework. VAE was applied to neural variational document model, which combines a continuous stochastic document representation with a bag-of-words generative model and achieves good results on both tasks [27]. The sequence-to-sequence model was trained with VAE for neural machine translation [28]. An extension of the recurrent neural network language models was proposed, which is designed to explicitly capture such global features in a continuous latent variable and applies KL-term annealing and input dropout techniques to improve training of VAE models [29]. A hierarchical latent variable RNN architecture was applied to the task of dialogue response generation, which facilitates both the generation of meaningful, long, and diverse responses and maintaining dialogue state [30]. A generative autoencoding sentence compression (ASC) model was proposed, which introduced a latent language model to provide the variable length compact summary [27]. A new generative model of sentences was addressed, which ﬁrst sampled a prototype sentence from the training corpus and then edited it into a new sentence and improved perplexity on language modeling and generated higher-quality outputs according to human evaluation [31].

## 3. Parse Tree Embedding VAE

The basic structure of our Tree-VAE contains two key modules: parse tree encoder module and VAE encoder-decoder module. A parse tree encoder is responsible for generating embedding vector of text structure. In VAE encoder-decoder module, a text encoder encodes the source text to a dense vector representation and a decoder generates realistic sentences from latent vector. The general architecture of Tree-VAE is shown in Figure 1. An encoder module is used to parse a tree and then train an encoder module based on the extracted structure information. The decoder can take a sentence as input and generate a text that contains multiple sentences of varying lengths and similar structures. The suggested technique necessitates that both modules have a basic degree of learning capacity.

### 3.1. Overview

The proposed approach contains two modules: a parse tree encoder module and a VAE encoder-decoder module. The parse tree encoder module ﬁrst extracts structural information content, and then the VAE encoder-decoder module is trained based on structural content. Given a sentence as input, the decoder can generate text, which contains multiple sentences of various lengths and similar structures. The proposed method requires the two modules to have initial learning ability. Therefore, we propose a pretraining method. The function of each module can be interpreted as follows. Syntax tree is more commonly used in theoretical syntax than parse tree in computational linguistics.

### 3.2. Parse Tree Encoder Module

The parse tree encoder module *E*_*θ*_ is used for explicitly extracting the structural information and feeding it into the VAE encoder-decoder module. We use a single Tree-LSTM [12] to generate the structural information of a sentence.

Given a source input sequence *x*=(*x*_1_, *x*_2_,…*x*_*T*_) of *T* words from Γ, the vocabulary of words, this module is responsible for producing a dense vector of structural content.  Figure 2 provides the overview of Tree-LSTM [12].

Since model learning requires the module with initial learning ability, we propose a pretraining method to teach the parse tree encoder module to effectively generate embedding vector for text structure. LSTMs perform far better when it comes to learning specific patterns. LSTM, like every other network, can have many hidden units, and as it goes through each level, the relevant information is retained, while the irrelevant data is eliminated in each cell. The resource that is responsible for creating a dense vector of structural content describes the incoming and outgoing sequences. Because model learning necessitates a module with initial learning ability, it effectively generates embedded vector for language structures. A syntactic parse tree-based similarity measure was used instead of RST measure. In the beginning, RST was developed as part of a study of computer-based text generation at MIT.

We construct a standard hierarchical LSTM network *D*_*ϕ*_ responsible for reconstructing the original structure tree based embedding vector and discard the hierarchical LSTM network when pretraining ends [13]. The motivation comes from the fact that, in a well-trained module, most structurally similar sentences have similar structural embedding vectors. The details are described as follows.

Given an input text sequence *x*, a structural parse tree *s* is produced as

(1) $$\begin{array}{c} s=\text{parser}\left(x\right). \end{array}$$

The parser employed is the standard dependency parser [10]. The text structure embedding vector *h* is computed as

(2) $$\begin{array}{c} h=E_{\theta }\left(s\right). \end{array}$$

In the above equation, *E*_*θ*_ is Tree-LSTM [12] network for parse tree encoder module, and *s* is text structure removed word content only keeping part of speech. We deﬁne *n*=(*n*_1_, *n*_2_,…*n*_*k*_) as the level order traversal result for tree *s*. *D*_*ϕ*_ is responsible for reconstructing sequence *n* based on embedding vector *h*. The cross-entropy loss is computed as

(3) $$\begin{array}{c} L_{\theta ,\phi }=-\sum_{ii=1}^{k}P_{D_{\phi }}\left(\frac{n_{i}}{h}\right),\\ =-\sum_{t=1}^{k}P_{D_{\phi }}\left(\frac{n_{i}}{E_{\theta }\left(s\right)}\right). \end{array}$$

### 3.3. VAE Encoder-Decoder Module

The standard VAE is a latent variable generative model, which combines variational inference with deep learning. Given a source input sequence *x*=(*x*_1_, *x*_2_,…*x*_*T*_), the encoder *Q*_*ψ*_ encodes input *x* into latent variable *z* with a posterior distribution *Q*_*ψ*_(*z|x*). Then the inputs are reconstructed by sampling *z* from this posterior and passing them through a decoder *G*_*ω*_. In order to make sampling easy, the posterior distribution is usually parametrized by a Gaussian with its mean and variance predicted by the encoder. The posterior *Q*_*ψ*_(*z|x*) is regularized with its KL divergence [14] from a prior distribution *p*(*z*). The loss is computed as

(4) $$\begin{array}{c} L_{\psi ,\omega }=-E_{z∼Q_{\psi }\left(z/x\right)}\left[\log\;P_{G_{\omega }}\left(\frac{x}{z}\right)\right]\\ +KL\left(Q_{\psi }\left(\frac{z}{x}\right)p\left(z\right)|\right). \end{array}$$

VAE has been viewed as a traditional autoencoder with some restrictions imposed on the internal representation space. In our work, the difference from that is that we train a VAE model conditioned on structure features *h* (provided by the parse tree encoder *E*_*θ*_). For the input sequence *x*, we ﬁrstly use pretrained parse tree encoder *E*_*θ*_ to generate text structure embedding vector *h* and then used encoder *Q*_*ϕ*_ encoding input *x* into the latent variable *z* and used decoder *G*_*ω*_ to reconstruct source text based on vector *h* and vector *z*. The loss is calculated as

(5) $$\begin{array}{c} L_{\psi ,\omega }=-Ez∼Q_{\omega }\left(\frac{z}{x,h}\right)\left[\log\;P_{G_{\omega }}\left(xz,h|\right)\right]\\ +KL\left(Q_{\psi }\left(z|x,h\right)|p\left(z\right)\right). \end{array}$$

Encoder *Q*_*ϕ*_ is only used for training and discarded at the test time. In the test stage, we ﬁrst sample a random prototype sentence *x* from the training corpus and then use *E*_*θ*_ to generate text structure embedding vector *h* and use to sample *z* for clarity of meaning and grammatical correctness. to sample *z* from this prior *p*(*z*); we ﬁnally use *G*_*ω*_(*x|z*, *h*) to output most structurally similar sentences. We implement *Q*_*ϕ*_ using two-layer LSTM network and implement *G*_*ω*_ using two-layer bidirectional LSTM network with attention. As a verb, “summarise” means to bring together the most important points of something; a summary is an example. It is called a conversational agent (CA) because it can converse with a human. A machine translation (MT) is a translation that is carried out automatically between languages. Machine translation has the advantage of being able to translate large amounts of text in a short amount of time. For those who order MT from us, it happens in a closed system via encrypted transmission. Expansion of VAE is vinyl acetate ethylene.

The details of the proposed Tree-VAE algorithm are shown in Algorithm 1. Overall, in the ﬁrst stage, we train a text structure information encoder *E*_*θ*_ and a text structure information decoder *D*_*ϕ*_. For a given sentence *x*, we generate a parse tree *s* by (1) and encode a parse tree *s* to a dense vector embedding *h* by Tree-LSTM. Then we optimize *E*_*θ*_ and *D*_*ϕ*_ based on the loss computed in (3). In the second stage, we train a condition text encoder *Q*_*ϕ*_ and a text decoder *G*_*ω*_ with VAE framework. For a given sentence *x*, we generate its structure embedding *h* by Tree-LSTM. Then we use *Q*_*ϕ*_ to compute the ﬁnal condition vector *z*. The decoder *G*_*ω*_ is responsible for generating text with ﬁnal condition vector *z*. We optimize *Q*_*ϕ*_ and *G*_*ω*_ based on the loss computed in (4).

## 4. Experiment

We evaluate our method on several real-world natural language generation tasks, review generation, speech language generation, and image captions generation.

### 4.1. Datasets

Three real-world public datasets are used in our research. Speech recognition is made easier with the help of a new language model built on recurrent neural networks.

  Yelp review corpus: This dataset is provided by Yelp^1^ (https://www.yelp.com/dataset). In our review generation experiment, the model accepts an input sentence and then generates an output sentence which likes input sentence. We randomly select 10000 sentences as the training set, select 2000 sentences as the validation set, and select 2000 sentences as the testing set, respectively.
  Email corpus: This dataset^2^ (https://www.kaggle.com/wcukierski/enron-email-dataset) contains approximately 500K emails generated by employees of the Enron Corporation. Like Yelp, we process this dataset by extracting a sentence that removed the last word as the source text and the sentences that removed the ﬁrst word as the target text. The processed dataset contains 170K, 80K, and 80K pairs for training, validation, and testing, respectively.
  COCO image captions corpus: It is provided by the COCO dataset [32]. The captions are the narrative sentences written by human, and each sentence consists of at least 8 words and at most 20 words. There are 5 captions per image. In each annotation, we take the ﬁrst sentence as the input text and the four following sentences as the target text. We randomly sample 1,800K, 500K, and 10K turns for training, validation, and testing, respectively. Two parts of the loss function exist: the reverse KL divergence and the loss function itself. Also note that the NN architecture of the encoder and decoder is of less importance than the NN architecture of the encoder.

### 4.2. Baselines

We compare our proposed method with the following baseline models:

  MLE: A standard sequence-to-sequence neural language model. To be fair, the settings of all sequence-to-sequence models are the same as those of our decoder.
  SVAE: The sentence variational autoencoder model [29].
  SeqGAN: A Sequence GAN that applied generative adversarial network with the policy gradient method and Monte Carlo (MC) search to text generation [33].
  RankGAN: A generative adversarial network for generating language descriptions. RankGAN trains the discriminator to learn and assign ranking scores, which helps to learn a better generator [19]. The complexity of JT-VAE is linear because it is a tree decomposition algorithm tailored for molecules, which has its roots in chemistry. Adhering to accepted standards of conduct or according to an accepted manner, model, or tradition.

### 4.3. Training Details

We set the hidden size to 256, embedding size to 128, and batch size to 64 for the parse tree encoder module and the VAE encoder-decoder module. We replace the nonfrequently used words (appeared less than 5 times) with the special character <UNK>. We use Adagrad optimizer with the initial learning rate of 0.1 [34]. For review generation, we set the number of generated sentences to 5, and the maximum length of each generated sentence is 30 words. For captions generation, we set the maximum length of each generated sentence to 20 words. In the parse tree encoder pretraining, the number of epochs is set to 100. In the VAE encoder-decoder module training, the number of epochs is set to 300. “Pretraining” refers to training a model with a single task to help it develop parameters that can be used in other tasks. People are the source of inspiration for pretraining, that is, initializing the model parameters of new tasks using the model parameters of previously learned tasks.

### 4.4. Experimental Results

#### 4.4.1. Automatic Evaluation

Following the evaluation protocol in [33], we calculate the BLEU score and estimate the similarity between the human-written text and the machine-generated text [35]. The key is to examine the similarity between the machine-generated findings and the human-provided references. The caption for this image is as follows: a popular artificial intelligence research area, generator is concerned with picture comprehension and a description of that image in a language. Syntactic and semantic knowledge of the language is required to construct well-formed sentences. Sequence-to-sequence models are a type of recurrent neural network architecture that we utilize (but are not limited to) to handle difficult language issues such as machine translation, question answering, chatbot creation, and text summarization (to name a few). Maximum Likelihood Estimation is a statistical technique that uses observed data to estimate the parameters of a probability distribution. Intuitive and flexible, the logic of maximum likelihood has become a standard method of statistical inference.

We use BLEU-2, BLEU-3, BLEU-4, and BLEU-5 to evaluate generation performance and use the whole test set as the references. “Tree-VAE (WA)” and “Tree-VAE (WOA)” represent Tree-VAE with attention mechanism and Tree-VAE without attention mechanism, respectively. From the results, it is obvious that the proposed model substantially outperforms the existing models, as shown in Table 1.

#### 4.4.2. Human Evaluation

We also conduct human study to evaluate the quality of the generated sentences. Each item contains 15 sentences written by different methods. The items are distributed to annotators who have no knowledge about which system the text is from. We require them to grade the generated text from 1 to 10 points considering relevance, diversity, and ﬂuency.  Table 2 shows the human evaluation scores. As we can see, when compared to language models, human-written phrases receive the best score. LTSM is an RNN model that can learn the problem of long-term dependence. Repeated modules chains make up recurrent neural networks in their purest form. It is a low-dimensional space into which high-dimensional vectors can be translated. This makes it easier to learn from large inputs such as sparse vectors of words. Learning and reusing embeddings are possible. In information theory, cross-entropy is an entropy-based measure of the difference between two probability distributions. A loss function based on cross-entropy can be used in the optimization of classification models like logistic regression or artificial neural networks.

#### 4.4.3. Analysis: Parse Tree Embedding

In this section, we provide detailed analysis to see the role of parse tree embedding. Object detection, segmentation, and captioning dataset COCO is a large-scale dataset for object detection, segmentation, and captioning. A bot is used for problems that do not require human intervention, such as those that do not require the use of both SeqGAN and RankGAN.

In Figure 3, we demonstrate the parse tree embedding distributions of some sampled sentences from true data. It can be seen that the parse embedding vector can reﬂect the structural similarity of text accurately. Embedding vector of sentences with similar structure is mapped to a 2-dimensional space with a closer distance. For example, as shown in the ﬁgure, “next the entire project goes on the balance sheet since we will be committed to building a road and stormwater system” and “the simpler way to bet on a potential rebound is with the shares of consumer and basic manufacturing companies near.” This white paper looks at how the memory types differ structurally and at performance analysis.

The two sentences, marked by circle, are sampled from the real data and the green point sentences near marked one are sampled from the most similar sentences with marked sentences (all real data are mapped to 2D space through the structure vector *h* with *pca*). It is important to note that the near sentences in vector space have very similar syntax structures. “Adagrad” stands for “Adaptive Gradient Algorithm” and it is an algorithm for optimizing gradients. Updates are made in small increments. Because of this, it works well with sparse data (NLP or image recognition). As each parameter learns at a different rate, it improves performance when dealing with problems involving sparse gradients. BLEU is a way to compare a generated sentence to one that has already been written in the target language. Score of 1.0 is awarded to perfect matches, and 0 is awarded to those that do not match perfectly.

We also compare the cosine structural similarity between real data parse tree embedding vector and generated data parse tree embedding vector. As presented in Figure 4, we calculate the mean cosine distance between each generated sentence and real test dataset, which reﬂects the structural rationality of the generated sentence. As we can see, the structure of sentences generated by Tree-VAE is more reasonable and the similarity with real data is much better than that of MLE. According to cross-entropy loss (or log loss), classification models that produce probabilities between zero and one perform poorly. As the projected probability differs from the labelled probability, the cross-entropy loss increases. It is just that as the predicted probability goes down, so too does the resulting log loss. Not all KL divergence is cross-entropy. For example, Kullback-Leibler divergence, or KL divergence, quantifies how much one distribution differs from another by measuring cross-entropy. KL divergence, in particular, measures a quantity very similar to cross-entropy.

Table 3 presents the examples generated by different models on the e-mail corpus dataset. We can find that these examples show that our model is able to generate more ﬂuent and novel sentences. The results show that our model can learn language generator effectively in a large corpus. It can be found that our model generates text with more higher diversity.

## 5. Conclusion

In this paper, we propose a novel model, called Tree-VAE, to promote the quality of the generated text. The Tree-VAE model used the structural features of a sentence as a condition for text generation, encouraging the decoder to produce coherent and meaningful text. In this framework, we adopted Tree-LSTM and Stanford Parser to extract sentences structures information and then train a conditional variational autoencoder generator condition on sentences structures embeddings. We evaluated the Tree-VAE on three datasets and the experiments showed that the Tree-VAE achieved excellent performance on generating sentences. In the future, we plan to explore and extend our model in many other tasks, such as image synthesis and dialogue system.

## Figures and Tables

**Figure 1:** Illustration of Tree-VAE. The parse tree encoder module extracts structural information from text. The encoder-decoder is based on the VAE trained over the real text condition on parse tree embedding vector.

**Figure 2:** The overview of Tree-LSTM. (a) A chain-structured LSTM network. (b) A tree-structured LSTM network with arbitrary branching factor.

**Figure 3:** Structural similarity between sentences.

**Figure 4:** Cosine similarity between embedding vectors *h* for true data and generated data of NLM and Tree-VAE.

**Algorithm 1:** Parse tree embedding VAE.

**Table 1:** Performance of the Tree-VAE and the four baselines on the Yelp review generation, e-mail generation, and COCO image captions generation tasks. Higher is better. “Tree-VAE (WA)” and “Tree-VAE (WOA)” represent Tree-VAE with attention mechanism and Tree-VAE without attention mechanism, respectively. BLEU-2, BLEU-3, BLEU-4, and BLEU-5 are the BLEU scores.

Yelp review	BLEU-2	BLEU-3	BLEU-4	BLEU-5

MLE	0.609	0.482	0.477	0.409
SVAE	0.663	0.654	0.587	0.571
SeqGAN	0.768	0.598	0.564	0.507
RankGAN	0.795	0.683	0.610	0.554
Tree-VAE (WA)	0.817	0.654	0.637	0.624
Tree-VAE (WOA)	0.806	0.697	0.664	0.631

E-mail	BLEU-2	BLEU-3	BLEU-4	BLEU-5

MLE	0.473	0.462	0.317	0.306
SVAE	0.548	0.517	0.441	0.353
SeqGAN	0.684	0.596	0.578	0.511
RankGAN	0.631	0.560	0.493	0.445
Tree-VAE (WA)	0.703	0.667	0.593	0.512
Tree-VAE (WOA)	0.711	0.670	0.600	0.527

COCO image captions	BLEU-2	BLEU-3	BLEU-4	BLEU-5

MLE	0.739	0.642	0.531	0.499
SVAE	0.801	0.784	0.668	0.633
SeqGAN	0.834	0.805	0.708	0.693
RankGAN	0.817	0.826	0.765	0.614
Tree-VAE (WA)	0.858	0.823	0.773	0.707
Tree-VAE (WOA)	0.853	0.819	0.794	0.730

**Table 2:** Results of human evaluation on three datasets. Higher is better.

	Model	Human score
Yelp	MLE	1.89
	SVAE	3.22
	SeqGAN	3.79
	RankGAN	3.83
	Tree-VAE (WA)	4.12
	Tree-VAE (WOA)	4.56

E-mail	MLE	2.03
	SVAE	2.55
	SeqGAN	3.72
	RankGAN	4.03
	Tree-VAE (WA)	4.41
	Tree-VAE (WOA)	4.63

COCO image captions	MLE	3.48
	SVAE	4.26
	SeqGAN	4.67
	RankGAN	4.55
	Tree-VAE (WA)	5.39
	Tree-VAE (WOA)	5.16

**Table 3:** Examples generated by Tree-VAE and baselines on the e-mail corpus dataset.

MLE:

sentence1: The company in this month<UNK>its earnings for the past four years.
sentence2: You might want to check to add value and differentiate in areas other than price to <UNK>going to them also.
sentence3: Just another update on where we have spent enough time.

SVAE:

sentence1: Phil have been invited to attend he web seminar at the system
sentence2: Gonzalez will be added to your shopping <UNK>and made the decision back up together.
sentence3: I expect complete important it by the close of additional databases.

SeqGAN:

sentence1: Follow the instructions to choose a new password
sentence2: We trust you will enjoy<UNK>our advertised companies.
sentence3: It works for works on both internal and external company e-mail on how to book this new opportunity.

RankGAN:

sentence1: We currently have two possible offers coming builder due to your strong local.
sentence2: I will get them signed and send them forward to discussing these meetings.
sentence3: I am very interested for people to pay the bills as soon as.

Tree-VAE:

sentence1: The followings are the folders that we use in the network drive for all existing computer.
sentence2: We found this to be the most effective and effective way to deal with tax issues.
sentence3: Last years, we were experiencing a major move, somany people played a key role in maintaining our team.

## Data Availability

The data used to support the findings of this study are available from the corresponding author upon request.
